The article "Residual Life Prediction of Lithium Batteries Based on Data Mining" was published in 2022. Journal: Comput Intell Neurosci.

# Residual Life Prediction of Lithium Batteries Based on Data Mining

**DOI:** 10.1155/2022/4520160

**Published:** 2022-06-13

**Authors:** Dandan Ma, Xiangge Qin

**Affiliations:** ^1^Information Science & Electronic Technology, Jiamusi University, Jiamusi 154007, Heilongjiang, China; ^2^Materials Science & Engineering, Jiamusi University, Jiamusi 154007, Heilongjiang, China

## Abstract

Lithium-ion batteries are an important part of smartphones, and their performance has a great impact on the life of the phone. The longevity of lithium-ion batteries is key to ensuring their reliability and extending their useful life. This paper built a lithium battery life prediction model and grey model MDGM(1,1) based on data mining. Then, experimental data were selected for testing, and the prediction error reached 10.5% at the minimum. It showed that the prediction model had higher precision and could provide help for the prediction and development of mobile phone battery life.

## 1. Introduction

With the advent of the era of “information explosion,” data mining arises at a historic moment to deal with the challenge of “knowledge shortage.” Data mining is a process of extracting valuable information and knowledge from a large amount of data. It has been widely used in society, economy, production, life, and other aspects. As we know, data mining is the massive historical data existing in databases, data warehouses, and external source files. However, some data have a small sample amount or are disabled, or the overall law is particularly complex, but the data in a certain time or space has strong regularity. At present, there is no effective data processing method, and the grey system theory can solve these problems very well. Taking advantage of grey system, it can be widely used in data mining. The two complementary advantages can make the discovered knowledge more effective and reliable.

Because of its advantages of lightweight, low discharge, and long life, lithium-ion battery is an energy storage device for portable electronics (such as notebook computers, digital cameras, tablet computers, mobile phones, and other handheld electronic products) [1]. As the core component of electronic products, in long-term use, due to various factors, the performance and life of lithium batteries will be affected, which may cause some troubles for users. That is why battery life has become a growing concern in recent years [2]. The basic composition of the battery pack is a single lithium battery. Therefore, the research of battery pack management system technology usually includes the monitoring of temperature, current and voltage of a single battery, capacity prediction, and charge state prediction of a single battery [3].

The article "Residual Life Prediction of Lithium Batteries Based on Data Mining" was published in 2022. Journal: Comput Intell Neurosci.

The research significance of this paper is mainly reflected in two aspects. Firstly, from the theoretical aspect, this paper combined the relevant theoretical data of data mining and grey system; at the same time, this paper also combines these two methods to establish the remaining life prediction model of lithium battery. Secondly, from the practical point of view, the lithium battery life prediction model constructed in this paper based on grey data mining can predict the life of lithium battery in advance and predict the battery life, which can effectively predict the future working ability of electronic products, timely find problems, and avoid unnecessary troubles and losses. This is very meaningful for the research and maintenance of lithium batteries.

## 2. Literature Review

### 2.1. Battery Life Prediction Technology

#### 2.1.1. Virtual Sample Technology

Traditional statistics are based on a sufficient sample number, but in reality, the sample number is limited or very small, which cannot meet the basic requirements of statistics. Therefore, a small sample is a classic problem [4]. In the era of big data, people are increasingly demanding for learning methods of two types of extreme sample data. These two types of sample data are massive samples that need to quickly obtain decision-making information due to big data and small samples that cannot obtain more data for learning in order to achieve fast response [5]. As the name implies, the problem of the small sample can be understood as the lack of information, but the key factors leading to the learning difficulty of the small sample are not all in the aspect of sample size. If there are a lot of data, but its distribution presents a discrete loose structure and there are gaps between sample points, the problem of incomplete and unbalanced samples will not be able to obtain effective information [6]. The problem of the small sample is mainly caused by unreasonable experimental design, high cost of obtaining sample data, or even the inability to obtain more sample data. In addition, it may also be due to the low probability of data occurrence, or although there are much data, it is data duplication. The problem of the small sample can be further divided into data scarcity, unbalanced data, and stability of feature selection of high-dimensional small sample [7]. High-quality data is the basis of effective decision-making. Therefore, to improve model-based accuracy and operability, it is an important work to expand the amount of effective data based on small sample data information to meet the requirements of modeling data.

The virtual sample is difficult to approximate the real sample completely and accurately. If too few virtual samples are generated, the additional information of unknown space carried by virtual samples is insufficient, and the generalization ability of the final model will be limited. If too many virtual samples are generated, on the one hand, the influence of real samples will be weakened, and on the other hand, errors introduced by virtual samples will deteriorate the generalization ability of the final model [8]. The more virtual samples are generated, the more untrusted information is brought in. Therefore, in order to maximize the generalization performance of the final model, there is an optimal number of virtual samples. The determination of the optimal virtual sample number has become an open problem in the research of the small sample problem [9].

The article "Residual Life Prediction of Lithium Batteries Based on Data Mining" was published in 2022. Journal: Comput Intell Neurosci.

#### 2.1.2. Battery Life Prediction

The capacity of a battery is an important indicator of battery performance, and its lifespan is an important indicator of its health. When the battery capacity decreases to a certain critical point (typically 80% of the rated capacity, but different battery types have different thresholds), the battery is considered to be invalid [10]. Remaining service life refers to the remaining service life of a battery after it has been used for a period of time [11–16]. For example, the power lithium battery has a cycle life of 500 times; that is, it can last 500 times under normal charging and discharging conditions. If it has been used 100 times, the remaining service life is 400 times. Generally, at present, the life prediction methods of lithium-ion batteries mainly include physical model and data-driven methods.

The physical model method mainly studies the internal structure of the lithium-ion battery and analyzes its physical and chemical changes. The formation of SEI film is considered to be the main cause of battery decay. The formation of SEI film consumes lithium ions inside the battery, and the internal resistance between electrode and electrolyte increases with the thickening of SEI film, which further leads to the decline of battery capacity [7, 17–19]. The method of the physical model involves the internal molecular level of the battery, which requires obtaining a large amount of information about the material properties and failure mechanism of lithium-ion batteries. However, internal chemical reactions are difficult to measure; it is difficult to predict the battery life through a physical model [12, 20]. The data-driven approach eliminates the need to study the internal chemical reactions of the battery and avoids the complex model of studying the interior of the battery, and on the basis of the existing experimental data, a functional model is obtained by using the method of data fitting [21–23]. Commonly used data-driven methods include grey model, BP neural network, SVM, correlation vector machine, ARMA model, and so on. The research object of this paper is the prediction of the remaining life of the lithium battery based on data-driven [24]. The capacity decay of lithium-ion batteries reflects the aging of batteries. Capacity refers to the amount of charge released in the complete process of discharging from full charge to empty charge, usually expressed in ampere-hour (Ah), as follows:

(1) $$\begin{array}{c} C=\int_{k}^{k+1}idt. \end{array}$$

When the current is constant, capacity C = It, where I represents the battery discharge current and T represents the discharge time. The capacity of the battery decreases with the life cycle of the battery. When the discharge capacity drops to 80%, it is considered to be the end of the service life. For example, when the battery power rating is 4 Ah, the aging threshold is 3.2 Ah. This paper uses experimental data to predict the capacity decay of the battery during charging and discharging cycles. [7].

The article "Residual Life Prediction of Lithium Batteries Based on Data Mining" was published in 2022. Journal: Comput Intell Neurosci.

### 2.2. Review of Lithium Battery Life Prediction

At present, although there are many kinds of lithium battery life prediction algorithms, according to the principle of modeling, it is divided into two types: physical model and data-driven. Each of these approaches is described below [14]. (1) Physical model-based methods refer to the prediction of remaining life (RUL) based on the physical properties of lithium batteries (e.g., material properties and loading conditions) and degradation mechanisms. (2) The data-driven RUL prediction method is to extract the characteristic parameters that can reflect the battery health status from the monitored variables such as voltage and current and build a statistical model of the system to extrapolate the prediction of RUL [25]. Because the data-driven method does not require the establishment of a complex system physical model, it is suitable for RUL prediction of complex and changeable internal lithium battery systems. Data-driven forecasting methods generally fall into two categories: artificial intelligence methods and statistics-driven methods [26].

Professor Deng Julong first proposed the grey theory in 1982. The theory is first applied in uncertain systems and then widely used in other systems. Its advantage is that it requires less data and has obvious advantages. The prediction methods based on grey theory include the metabolic Markov residual grey model and metabolic grey model. By selecting different models under different conditions, the applicability of the models is improved, and the estimation accuracy is also improved [27].

The article "Residual Life Prediction of Lithium Batteries Based on Data Mining" was published in 2022. Journal: Comput Intell Neurosci.

According to the principle of non-equilibrium thermodynamics, Virkar built a degradation mechanism model of the lithium battery by analyzing the electrochemical reaction inside the battery and added SEI membrane and chemical potential into the process of predicting RUL. Gong has proposed a method for predicting the residual life of lithium batteries based on a gas generation model.

According to the analysis and research on the actual gas generation mechanism of the battery, the types of chemical reactions in the battery were determined, and the gas generation equation was established. Based on these gas equations, a relationship model between battery capacity and gas production characteristics was established, and a prediction model for the remaining life of lithium battery was established finally. TPF is a probability density function represented by random samples in the state space [28, 29].

To sum up, the fusion model-based method is still the focus of future research. It not only improves the prediction accuracy but also improves the robustness of model output. However, its disadvantages are high algorithm complexity and large computation. In addition, most of the research on battery life prediction are still in the laboratory stage, so it is still a long way to go.

## 3. Lithium Battery Life Prediction Model Construction Based on Data Mining

### 3.1. Grey Data Mining System

The grey data mining system draws on the structure of the traditional data mining system and makes full use of the grey system method to carry out data mining. It is based on a database and data warehouse and provides effective methods for data mining tools of data warehouse [16].  Figure 1 shows the system architecture.

### 3.2. Establishment of Grey Model MDGM(1,1)

Since it was proposed by Deng Julong in 1982, the grey system has been widely used in various forecasting fields. Metabolism discrete grey prediction MDGM(1,1) model is the core of grey system theory. MDGM(1,1) quantifies the abstract concept of the known information in the system first, then processes the quantified concept through modeling, and finally optimizes the model to predict the unknown data. Grey prediction MDGM(1,1) model has long been concerned and valued by people.

The MDGM(1,1) model is formed by the first-order differential equation with only one variable. First of all, the original sequence is accumulated and generated to present a certain rule; then the first-order linear differential equation model is established; and finally, the fitting curve is obtained to predict the system, which is the process of establishing MDGM(1,1) model. Details are as follows:

Let *X* (0) be a nonnegative sequence:

(2) $$\begin{array}{c} X^{\left(0\right)}=\left(X^{\left(0\right)}\left(1\right),X^{\left(0\right)}\left(2\right),\ldots ,X^{\left(0\right)}\left(n\right)\right). \end{array}$$

First-order accumulation is

(3) $$\begin{array}{c} X^{\left(1\right)}=\left(X^{\left(1\right)}\left(1\right),X^{\left(1\right)}\left(2\right),\ldots ,X^{\left(1\right)}\left(n\right)\right). \end{array}$$

Adjacent to the mean-generating sequence

(4) $$\begin{array}{c} Z\left(1\right)=Z^{\left(1\right)}\left(2\right),Z^{\left(1\right)}\left(3\right),\ldots Z^{\left(1\right)}\left(n\right) \end{array}$$

if

(5) $$\begin{array}{c} \hat{a}={\left[a,b\right]}^{T}. \end{array}$$

The GM(1,1) model is

(6) $$\begin{array}{c} X^{\left(0\right)}\left(k\right)+aZZ^{\left(1\right)}\left(k\right)=b. \end{array}$$

The least-square estimation parameter column satisfies

(7) $$\begin{array}{c} \hat{a}={\left[B^{T},B\right]}^{-1}B^{T}Y \end{array}$$

if the set is

(8) $$\begin{array}{c} X^{\left(0\right)}\left(k\right)=\left(\beta -aX^{\left(0\right)}\left(1\right)\right)e^{-a\left(k-2\right)}. \end{array}$$

The above equation is the basis for prediction in this paper.

The article "Residual Life Prediction of Lithium Batteries Based on Data Mining" was published in 2022. Journal: Comput Intell Neurosci.

### 3.3. Accuracy Test of Grey Model MDGM(1,1)

After calculation, the small error probability *p* is 0.983; the ratio of post-test square difference C is 0.251; and the accuracy level is 1; and it shows that the model can be used for prediction. The grey GM(1,1) model is used to predict the life of lithium-ion batteries, as shown in Figure 2.

According to Figure 2, Battery18 reaches the failure point after 100 cycles of charging and discharging, so its real life is 100 cycles. When the starting point of prediction is 60 cycles, the life failure point predicted by the grey GM(1, 1) model is 120 cycles. The error is 20 cycles; the prediction accuracy is ordinary; for the convenience of comparison, the predicted results at *T* = 40, 60, and 80 cycles were put on the same graph, as shown in Figure 3.

To sum up, GM(1,1) model in grey theory is used to predict the life of the lithium-ion battery in this section. The experimental results show that the prediction effect of this method is acceptable, but the accuracy needs to be improved. As the capacity decay trajectory of the lithium-ion battery is nonlinear and random, the predicted trajectory of the grey model is close to a straight line, which can be regarded as the prediction of the trend term in the capacity degradation trajectory, but the random term is not predicted. Considering the degradation of battery capacity can also be regarded as a series of time series, the life prediction of the lithium-ion battery can be further studied by time series analysis.

The article "Residual Life Prediction of Lithium Batteries Based on Data Mining" was published in 2022. Journal: Comput Intell Neurosci.

As an important grey theory, the grey prediction method is widely used in the engineering field. Sun Tao et al. applied the grey system theory to the project cost and established the grey model to realize the estimate of the project cost with high precision. Xu hui et al. conducted a grey correlation analysis on the measured data of the dam and established the GM(1,1) model to predict the dam settlement on this basis. The results show that the method is effective. Li Peng and others. Based on the improvement of the traditional GM(1, 1) model, the grey relational model of GM(1, *N*) is put forward and applied to the capacity prediction of lead-acid batteries. Gu Weijun and so on. In view of the small sample of battery life data and the long test of battery life, the grey GM(1, 1) model is used to predict the cycle times when the battery reaches the specified life end value to estimate the battery lifetime.

## 4. Test Results and Analysis

### 4.1. Battery Capacity Degradation Data Analysis

Prediction is to estimate the future state of a product based on its past state of change. Specifically, RUL prediction mainly refers to the estimation of the remaining time from the current time to the final failure according to the monitored historical data of the product itself or similar products when the product runs to moment *i* (time here refers to the generalized time). Among them, historical data can be status monitoring data, failure time, maintenance time, or other event data. Given the status monitoring data of a product up to the current moment *T*, the method based on artificial intelligence is further subdivided into the statistical regression method and the similarity method.

Statistical data-driven RUL prediction methods can be divided into direct monitoring data-based RUL prediction method and indirect monitoring data-based RUL prediction method from the perspective of state monitoring data type. Direct state monitoring data is essentially the deterioration data of products. However, the literature does not consider the RUL prediction method combined with the historical data of similar products. This section summarizes the relevant RUL prediction methods from the perspective of degradation data, analyzes the advantages and disadvantages of each method, and discusses some problems worthy of study. Therefore, in this paper, the curve-grey model is used to analyze and predict the capacity degradation data, and the data are used to verify the model algorithm.

Using the grey mathematical model, a mathematical model of the capacity decay of lithium-ion batteries under constant current discharge, constant temperature, and constant depth of discharge is established. B5, B6, and B18 batteries were selected as samples to verify the model and algorithm. The discharge currents of B5, B6, and B18 batteries were all 2 A, and the three batteries carried out 168, 168, and 132 charge and discharge cycles, respectively, with discharge voltages of 2.7 V, 2.5 V, and 2.5 V.

The article "Residual Life Prediction of Lithium Batteries Based on Data Mining" was published in 2022. Journal: Comput Intell Neurosci.

As can be seen from Figures 4–6, the capacity of a single lithium-ion battery decreases gradually with the increase of charge and discharge cycles. Among them, B5 and B6 show an obvious linear decline trend, while B18 (after different processing) shows an exponential degradation trend during the first 10 charge and discharge cycles and then shows a linear degradation trend.

### 4.2. Analysis of Test Methods

In order to verify the performance of the mobile phone battery life prediction algorithm and prove its effectiveness, experimental data of different types of batteries under different experimental conditions would be selected in this paper for experimental analysis and evaluation of the grey data mining model construction method.

1. Firstly, using the measured data of four lithium-ion batteries of NASA, the relationship between constant discharge voltage and battery capacity before and after Box-Cox conversion is analyzed, and the relationship between Box-Cox conversion parameters is also studied. And, based on GM(1, 1), the effectiveness and correctness of the method are verified by comparison.
2. Secondly, in order to verify the adaptability of the method, the battery test data of the GM(1,1) model is used to verify the adaptability of the method. In order to fully verify the performance of the proposed method throughout the experiment, the data of equal discharge voltage difference at three time intervals were used for experimental verification of each battery.

### 4.3. Analysis of Test Results

#### 4.3.1. Grey Model Prediction Process

The following is the process for predicting the remaining life of lithium-ion batteries using the GM(1, 1) model.

**Step 1 .**

Original data of lithium-ion capacity degradation assuming cyclic charging and discharge is C = {Ci, I = 1, 2,…, N}, and the original data are, respectively, accumulated once:

(9) $$\begin{array}{c} C_{i}^{\left(1\right)}\left(k\right)=\sum_{i=1}^{k}C_{i},\;i=1,2,\ldots ,k. \end{array}$$

Get a summation-generated sequence vector.

**Step 2 .**

Identify the unknown parameters in the model. Calculate the background value of the GM(1,1) model as follows:

(10) $$\begin{array}{c} Z\left(k\right)=0.5\times \left(C_{K}^{\left(1\right)}+C_{K-1}^{\left(1\right)}\right). \end{array}$$

The function expression of GM(1,1) is

(11) $$\begin{array}{c} \frac{dc_{i}^{\left(1\right)}}{dt}+aC_{i}^{\left(1\right)}=b. \end{array}$$

For the first-order grey model GM(1,1), the following equation can be obtained:

(12) $$\begin{array}{c} B_{N}a=Y_{N}. \end{array}$$

**Step 3 .**

The article "Residual Life Prediction of Lithium Batteries Based on Data Mining" was published in 2022. Journal: Comput Intell Neurosci.

Solve the GM(1,1) model. The time response vector is

(13) $$\begin{array}{c} C_{i}^{\left(1\right)}=\left(C_{0}^{\left(1\right)}-\frac{b}{a}\right)\text{exp}\left(-at\right)+\frac{b}{a}. \end{array}$$

**Step 4 .**

Predict the remaining service life of the lithium-ion battery through the established grey model.

The capacity degradation model of the lithium-ion battery can be expressed as follows:

(14) $$\begin{array}{c} {\hat{C}}_{N+P}=\left(C_{1}-\frac{{\hat{b}}_{N}}{{\hat{a}}_{N}}\exp\left(-{\text{a}}_{N}\left(N+P\right)\right)\right)\exp\left({\hat{-a}}_{N}-1\right). \end{array}$$

Also, the prediction accuracy of the proposed method was evaluated according to the relative error of the remaining service life prediction of lithium-ion batteries as follows:

(15) $$\begin{array}{c} \text{RUL error}=\frac{\left(\text{RUL tuue}-\text{RUL prediction}\right)}{\text{RUL true}}. \end{array}$$

#### 4.3.2. Prediction Effect of the Discrete Grey Model

The following is an introduction to the feasibility of using NASA data to validate the grey model to predict lithium-ion battery RULs. Select the capacity degradation data for B6 and B18. The training data of the first 70 times, and the first 80 times were selected, and the failure threshold was set to 80%. Figures 7 and 8 show the battery prediction results.

The feasibility of the algorithm using NASA data is shown below. B6 and B18 battery capacity degradation data are selected. The first 70 and 80 times of training data are selected, and the failure threshold is set to 80%. The prediction errors obtained are shown in Table 1.

## 5. Conclusion

Aiming at the life prediction of the lithium-ion battery in smartphone, a life prediction method based on grey data mining model is proposed, and the proposed method is verified and evaluated. In this paper, data mining and grey system theory are studied. Grey MDGM(1, 1) model is used as the life prediction method of the lithium-ion battery. Based on the above method, a grey data mining model is proposed to predict the degradation trajectory of lithium-ion batteries, which is nonlinear and random. The grey MDGM(1, 1) model has been used to describe the trend items in the degradation data to further improve the prediction accuracy. The battery test data for NASA PCoE is used to validate the model.

Due to the influence of time and equipment conditions, the research on the life prediction of lithium-ion batteries of smartphones in this paper is not sufficient. There are still the following problems, which need to be further improved in the future work:

1. In this paper, the life prediction methods of lithium-ion batteries are all about a single lithium-ion battery, while batteries in mobile phones are often in the form of battery packs, so battery packs should be considered in the future.
2. The data used in this paper are all obtained under the experimental conditions of constant current and constant voltage, while the actual working conditions of lithium-ion batteries on mobile phones are very complicated. Different charging and discharging mechanisms and different environments will affect its capacity degradation process. Therefore, capacity degradation data under different charging and discharging mechanisms should be used to verify the model in the future.

The article "Residual Life Prediction of Lithium Batteries Based on Data Mining" was published in 2022. Journal: Comput Intell Neurosci.

## Figures and Tables

**Figure 1:** Structure of the grey data mining system.

**Figure 2:** Prediction results of lithium-ion battery life based on grey model.

**Figure 3:** Life prediction of lithium-ion battery based on grey model (B18).

**Figure 4:** Capacity degradation of the B5 lithium battery.

**Figure 5:** B6 lithium battery capacity degradation data.

**Figure 6:** B18 lithium battery capacity degradation data.

**Figure 7:** Battery prediction result (the first 70 volume data).

**Figure 8:** Battery prediction result (the first 80 volume data).

**Table 1:** Prediction errors.

Training data	The actual	RUL to predict	Error (%)
70	105	89	17.9
80	105	88	19.3

## Data Availability

The data set can be obtained from the corresponding author upon request.
